The article "PITX2 enhances progression of lung adenocarcinoma by transcriptionally regulating WNT3A and activating Wnt/β-catenin signaling pathway" was published in 2019. Journal: Cancer Cell Int.

# PITX2 enhances progression of lung adenocarcinoma by transcriptionally regulating WNT3A and activating Wnt/β-catenin signaling pathway

**DOI:** 10.1186/s12935-019-0800-7

**Published:** 2019-04-11

**Authors:** Jing Luo, Yu Yao, Saiguang Ji, Qi Sun, Yang Xu, Kaichao Liu, Qiang Diao, Yong Qiang, Yi Shen

**Affiliations:** 1 Department of Cardiothoracic Surgery, Jinling Hospital, 305 East Zhongshan Road, Nanjing, China; 2 Jiangsu Key Laboratory of Molecular and Translational Cancer Research, Nanjing, China; 3 Department of Respiratory Medicine, Nanjing Second Hospital, Medical School of Southeast University, Nanjing, China; 4 Bengbu Medical College, Bengbu, Anhui China; 5 Department of Medical Imaging, Jinling Hospital, 305 East Zhongshan Road, Nanjing, China

**Keywords:** PITX2, Lung adenocarcinoma, Wnt/β-catenin, miR-140-5p

## Abstract

**Background:**

The homeodomain transcription factor, PITX2 is associated with tumorigenesis of multiple cancers. In this research, we aimed to study the expression, function and mechanism of PITX2 in lung adenocarcinoma (LUAD).

**Methods:**

The TCGA dataset was used to analyze the expression and clinical significance of PITX2 in LUAD. The expression of PITX2 in tumor samples and LUAD cell lines was examined by quantitative real-time PCR (qRT-PCR) and western blotting. Small interfering RNAs (siRNAs) were constructed to knockdown PITX2 and to determine the physiological function of PITX2 in vitro. Xenograft model was used to confirm the role of PITX2 in vivo.

**Results:**

PITX2 was overexpressed in LUAD and patients with high level of PITX2 had a worse overall survival and an advanced clinical stage. Knockdown of PITX2 inhibited cell proliferation, migration and invasion of LUAD cells. Further study revealed that the oncogenic role of PITX2 was dependent on activating Wnt/β-catenin signaling pathway, especially by transcriptionally regulating the Wnt gene family member, WNT3A. Lastly, we identified miR-140-5p as a negative mediator of PITX2 by binding its 3′UTR and ectopic expression of miR-140-5p inhibited progression of LUAD cells via suppressing the expression of PITX2.

**Conclusions:**

Up-regulation of PITX2 acts as an oncogene in LUAD by activating Wnt/β-catenin signaling pathway, suggesting that PITX2 may serve as a novel diagnostic and prognostic biomarker in LUAD.

**Electronic supplementary material:**

The online version of this article (10.1186/s12935-019-0800-7) contains supplementary material, which is available to authorized users.

## Background

Lung adenocarcinoma (LUAD) is the most common histologic subtype of lung cancer, with an increasing morbidity and mortality rate over the past decades [1, 2]. Multiple genomic alterations are discovered to be associated with the progression of LUAD and significant advances have been achieved in molecularly targeted therapy [3]. However, drug resistance and side effects weaken the therapeutic effects and the overall 5-year survival rate of LUAD is still less than 20% [4]. Thus, a further understanding of the cellular mechanisms that regulate LUAD progression may provide alternative diagnostic markers and therapeutic targets for LUAD patients.

The article "PITX2 enhances progression of lung adenocarcinoma by transcriptionally regulating WNT3A and activating Wnt/β-catenin signaling pathway" was published in 2019. Journal: Cancer Cell Int.

The homeobox genes are a group of genes containing homeobox (a 180 base pairs long DNA sequence) and encode homeodomain proteins that act as transcription factors [5]. Many homeobox genes have been proved to be implicated in various human cancers, acting as oncogenes or tumor suppressors [6–8]. Paired-like homeodomain transcription factor 2 (PITX2), a member of the bicoid/paired-like homeobox gene family, is located on chromosome 4q25 and encodes a transcription factor involved in the development of anterior structures [9, 10]. Recent studies have highlighted the association of PITX2 with progression of many human cancers, including gonadotroph tumor, colorectal cancer, thyroid cancer and esophageal squamous cell carcinoma [11–14]. However, the expression of PITX2 in LUAD and its effect on biological behavior of LUAD have not been elucidated.

Earlier researches have discovered that homeobox genes are actively involved in the regulation of the Wnt pathway [15–17]. Particularly, PITX2 is reported to regulate the Wnt/β-catenin pathway by activating Wnt ligand genes and thus contributing to cancer progression [18]. The Wnt/β-catenin signaling pathway was first identified for its role in carcinogenesis and meanwhile it was confirmed to be essential for embryonic development [19, 20]. Herein we investigated the influence of PITX2 on activity of Wnt/β-catenin pathway in LUAD.

MiRNAs, a class of 18–25 nucleotide non-coding RNAs, have emerged as key regulators of gene expression at the post-translational level by combining with the 3′UTRs (untranslated regions) of their target mRNAs [21]. The miRNA-mediated gene post-transcriptional regulation is involved in various aspects of physiological processes [22]. And studies are increasingly implicating miRNAs in the progression of many types of cancer, including LUAD [23–25]. Since the regulatory miRNAs could suppress target mRNAs and play a critical role in pathogenesis, we performed experiments to determine whether PITX2 is targeted by specific miRNA.

## Materials and methods

### Bioinformatics

To determine the expression of PITX2 in LUAD and normal lung tissues, the TCGA dataset named TCGA_LUAD_exp_Hi-SeqV2-2015-02-24, were downloaded from the UCSC Cancer Browser (https://genomecancer.ucsc.edu/) [26]. The “genomicMatrix” file was browsed to get the normalized expression of PITX2 in LUAD and the clinicopathological information of patients was acquired from “clinical_data” file. The cBioPortal website (http://www.cbioportal.org/) [27] was used to obtain highly co-expressed genes with PITX2. Totally 317 genes (Additional file 1: Table S1) were submitted to DAVID Bioinformatics Resources 6.8 (http://david.abcc.ncifcrf.gov/) [28] and Reactome Pathway Database (https://reactome.org/) [29] for Gene_Ontology pathway and Reactome pathway analysis, respectively. The protein association networks of PITX2 were derived from The String Database (https://string-db.org/) [30]. The transcription factor binding site (TFBS) of PITX2 was exhibited in Human Transcription Factor Database Version3.0 (http://bioinfo.life.hust.edu.cn/AnimalTFDB/#!/) [31] and hTFtarget database (http://bioinfo.life.hust.edu.cn/hTFtarget#!/) was utilized to analyze the potential binding site of PITX2 with target genes. To search for miRNAs that directly target PITX2, CoMeTa dataset (http://cometa.tigem.it/index.php) [32], DIANA lab tools webpage (http://diana.imis.athena-innovation.gr/DianaTools/index.php?r=site/index) [33] and the microRNA database (http://www.microrna.org/microrna/home.do) [34] were used.

The article "PITX2 enhances progression of lung adenocarcinoma by transcriptionally regulating WNT3A and activating Wnt/β-catenin signaling pathway" was published in 2019. Journal: Cancer Cell Int.

### Patient tissue samples

60 pairs of LUAD tissues were obtained from patients who had undergone radical surgical resection in the department of thoracic surgery, Nanjing Jinling Hospital. All tissues were examined by two experienced pathologists who confirmed the TNM stage of each patient. The clinical information of patients was consulted from their medical records. And the study was approved by Ethics Committee of Nanjing Jinling Hospital and informed consent was obtained from all patients.

### RNA extraction, reverse transcription, and qRT-PCR

Total RNA of tissue or cell samples were extracted with TRIzol Reagent (Invitrogen). The extracted RNA was dissolved with RNAase-free water, and 1.5 μg RNA from each sample was used for cDNA synthesis using a Reverse Transcription Kit (Takara, cat: RR036A). SYBR Select Master Mix (Applied Biosystems, Cat: 4472908) was used for qRT-PCR and primers are shown in Additional file 2: Table S2. The comparative C_T_ method (ΔΔC_T_) was used to measure the relative gene expression.

### Immunohistochemistry (IHC)

Paraffin-embedded sections were deparaffinized and incubated in retrieval buffer solution for antigen retrieval. The sections were incubated with corresponding antibodies: anti-PITX2 (Sigma-Aldrich, AV35634, 1:100), anti-WNT3A (Abcam, ab28472, 1:100), anti-CyclinD1 (Cell Signaling Technology, 2978, 1:100), anti-C-Myc (R&D Systems, AF3696, 1:100).

The article "PITX2 enhances progression of lung adenocarcinoma by transcriptionally regulating WNT3A and activating Wnt/β-catenin signaling pathway" was published in 2019. Journal: Cancer Cell Int.

### Cell lines and cell culture

LUAD cell lines (NCIH1975, NCIH1650, PC9, A549, NCIH1299) and human bronchial epithelial cell (HBE) were purchased from Shanghai Institutes for Biological Science, China. NCIH1975, NCIH1650 and HBE cells were cultured in DMEM medium (KeyGene), and PC9, A549 and NCI-H1299 cells were cultured in RPMI 1640 medium (KeyGene), supplemented with 10% fetal bovine serum. All cells were cultured at 37 °C in a humidified incubator containing 5% CO_2_.

### Western blotting

Western blotting was performed according to standard protocols as previously described [35]. Briefly, cultured cells were lysed with lysis buffer (RIPA, KeyGEN) containing protease inhibitors (PMSF, KeyGEN) on ice, and protein concentration was determined using a BCA Kit (KeyGEN). Western blotting were obtained utilizing 30 μg of lysate protein. The antibodies used were as follows: anti-β-actin (Cell Signaling Technology, 3700, 1:1000), anti-PITX2 (Abcam, ab55599, 1:1000), anti-CyclinD1 (Cell Signaling Technology, 2978, 1:1000), anti-CD44 (Cell Signaling Technology, 3570, 1:1000), anti-C-Myc (R&D Systems, AF3696, 1:1000), anti-C-Jun (Cell Signaling Technology, 9165, 1:1000), anti-WNT3A (Abcam, ab28472, 1:100).

### Transfection

siRNAs against PITX2 (Santa Cruz Biotechnology, sc-44016) were used at 20 nM/well using 2 μL Lipofectamine RNAiMAX (Invitrogen) in the cells seeded in 6-well plates. The full-length cDNA of human PITX2 were PCR-amplified and cloned into the expression vector pENTER (Vigene Biosciences). shRNA and microRNA mimics were conducted and purchased from Vigene Biosciences. Transfection of plasmids and miRNA mimics was performed according to the Lipofectamine 3000 Reagent (Invitrogen) protocol. Totally 10 μg plasmid vectors were transfected into cells seeded in 6-well plates for each group. Nonsense shRNA (sh-nc) and negative control mimics were used as the respective controls. The sequences of shRNAs and microRNA mimics are shown in Additional file 3: Table S3.

### Cell proliferation assay

For the Cell Counting Kit-8 (CCK-8) assay, cells were plated in 96-well plates at a density of 4000 cells/100 μL, and the absorbance was measured at 450 nm in an ELx-800 Universal Microplate Reader. Real time xCELLigence system (RTCA) assay was performed according to the instructions provided by the manufacturer [36]. And cells were placed in 6-well plates at 400 cells per well for colony formation assays. After 10–14 days, the cells were fixed using 4% paraformaldehyde and stained with 0.1% crystal violet solution.

### Migration and invasion assay

Transwell assay inserts (8 μM PET, 24-well Millicell) or Matrigel-coated membranes (BD Biosciences) were add with 200 μL serum-free medium in the upper chamber and 800 μL serum-containing medium in the lower chamber. Totally 50,000 cells were added to the upper chamber and cells in lower chamber were fixed and stained after 24 h (migration) or 48 h (invasion).

The article "PITX2 enhances progression of lung adenocarcinoma by transcriptionally regulating WNT3A and activating Wnt/β-catenin signaling pathway" was published in 2019. Journal: Cancer Cell Int.

### Flow cytometry assay

Flow-cytometry analysis was performed to detect cell cycle distribution. Cells were harvested after transfection with siRNA for 48 h and fixed in 1 mL 70% ethanol at − 20 °C. The ethanol-suspended cells were centrifuged and stained with PI staining solution for 10 min in the dark at 37 °C. A FACSCalibur flow cytometer was used to detect cell cycle distribution. The percentage of cells in G1, S, and G2-M phases were counted and compared.

### TUNEL (TdT-mediated dUTP nick-end labeling) assay

TUNEL Kits (KeyGEN BioTECH, KGA7062) were used to detect DNA fragmentation of apoptotic cells. Cells were seeded in 24-well plates and fixed with 4% paraformaldehyde. After washing with PBS and 0.5% Triton X-100, cells were incubated at 37 °C for 1 h from light with terminal deoxynucleotidyl transferase enzyme and cell nuclei were counterstained with DAPI. Images were obtained from a fluorescence microscope and apoptosis ratio was calculated.

### Luciferase reporter assay

The WNT3A promoter region (− 2000 bp) or PITX2 3′UTR was amplified and cloned into luciferase reporter plasmid (pGL3-basic). The luciferase reporter plasmids were co-transfected with CMV-PITX2 expression plasmids or miRNA mimics. And CMV-empty vector or miRNA control mimics were used as negative controls. CMV-Renilla was used as an internal control and Firefly/Renilla value was used to measure luciferase activity. After transfection for 48 h, cells were harvested and assessed for luciferase activity using the Dual Luciferase Reporter Assay System (Promega).

### ChIP (chromatin immunoprecipitation) assay

Cells were cross-linked in 4% paraformaldehyde and the reaction was quenched with 10× glycine. Then cells were added with pre-cooling PBS (containing 5 μL protease inhibitor, cocktail) and scraped into a centrifuge tube, followed by centrifuging for 10 min at 800×*g* at 4 °C. Cell precipitates were resuspended in 500 μL cell lysis buffer (containing 2.5 μL cocktail) and 500 μL nucleus lysis buffer (containing 2.5 μL cocktail) successively. After that, the cells were sonicated (amplitude 30%) on ice to break DNA into fragments and were centrifuged for 10 min at 12,000*g* at 4 °C. For immunoprecipitation, the above products were added with 5 μg anti-PITX2 antibody (Abcam, ab192495) or 5 μg mouse IgG (Santa Cruz Biotechnology, sc-2025), all of which were mixed with 100 μL Dilution buffer and 20 μL magnetic beads (Resin M2, Sigma), and then incubated at 4 °C overnight. For DNA purification, immunoprecipitation products were added with ChIP elution buffer (containing proteinase K) and then was heated at 62 °C for 2 h and 95 °C for 10 min. Finally, the DNA was eluted with elution buffer in adsorption column and used for PCR reaction. The sequence of primers used are shown in Additional file 2: Table S2 and GAPDH was used as a control.

The article "PITX2 enhances progression of lung adenocarcinoma by transcriptionally regulating WNT3A and activating Wnt/β-catenin signaling pathway" was published in 2019. Journal: Cancer Cell Int.

### Animal studies

LUAD tumor cells were transfected with shRNAs or control plasmids before transplantation. Six female nude mice (4–6 weeks old) per group were purchased from Nanjing Medical University School of Medicine’s accredited animal facility. 2 × 10^6^ LUAD tumor cells in 100 μL sterile PBS were injected subcutaneously to each mouse and tumors were harvested at 6 weeks after injection. The weight of tumor was measured on the scale and tumor volume was estimated using calipers ([length * width^2^]/2). And the tumor tissues were immunohistochemically stained with corresponding antibodies. All animal studies were conducted in accordance with NIH animal use guidelines and protocols were approved by Nanjing Medical University Animal Care Committee.

### Statistical analysis

Generally experiments were repeated for three times and data were presented as the mean ± SD. Student’s *t* test was used to assess the differences between two groups. Chi square test was performed to analyze the differences between variables. Bivariate correlations between study variables were calculated by Pearson’s correlation coefficients. Kaplan–Meier method was used to plot survival curves. Statistical analysis was performed using SPSS Statistics software (version 20.0). p < 0.05 was considered statistically significant. Graphs were made using the GraphPad Prism 6.0 software package.

## Results

### PITX2 was overexpressed in LUAD and correlated with worse prognosis

By analyzing the TCGA dataset (TCGA_LUAD_exp_Hi-SeqV2-2015-02-24), the expression of PITX2 was upregulated in LUAD tissues (n = 511) compared with normal tissues (n = 58) (Fig. 1a). And for the 511 LUAD tissues included in TCGA dataset, patients with higher PITX2 expression (the upper quartile, n = 128) had a more dismal overall survival than those with lower PITX2 expression (the lower quartile, n = 128) (Fig. 1b). The Chi squared test suggested that the PITX2 level is also related to T stage (p = 0.00311), M stage (p = 0.0367) and TNM stage (p = 0.010652) (Table 1). For further verification, we examined the levels of PITX2 in 60 pairs of LUAD and non-tumor tissues collected from Department of Cardiothoracic Surgery, Jinling Hospital. The results showed that PITX2 was upregulated in 76.67% of LUAD tissues (Fig. 1c). The clinical data of these patients was shown in Additional file 4: Table S4. Unpaired t test was used to validate the correlation between PITX2 and clinical pathological characteristics. The expression of PITX2 in patients of stage T2 (7.116 ± 1.130, N = 27), T3 (15.51 ± 3.166, N = 6) and T4 (20.54 ± 6.943, N = 4) was higher than patients of stage T1 (3.430 ± 0.8230, N = 23) (Fig. 1d). And patients with lymph node metastasis (14.05 ± 3.054, N = 12) had a higher PITX2 expression than patients without lymph node metastasis (5.783 ± 0.8629, N = 48) (Fig. 1e). Moreover, patients of TNM stage II (11.63 ± 1.179, N = 25) and III (16.55 ± 6.693, N = 5) had a higher PITX2 expression than patients of stage I (2.427 ± 0.5142, N = 30) (Fig. 1f). In addition, the mRNA and protein level of PITX2 were elevated in LUAD cell lines (NCIH1975, NCIH1650, PC9, A549, NCIH1299) compared with Human Bronchial Epithelial (HBE) Cells (Fig. 1g, h). The data suggested that PITX2 was a potential upregulated oncogene in LUAD.

The article "PITX2 enhances progression of lung adenocarcinoma by transcriptionally regulating WNT3A and activating Wnt/β-catenin signaling pathway" was published in 2019. Journal: Cancer Cell Int.

**Fig. 1:** PITX2 was highly expressed in lung adenocarcinoma and correlated with clinicopathological characteristics. **a** Utilizing the TCGA dataset, we found that PITX2 was overexpressed in lung adenocarcinoma compared with adjacent normal tissues (Normal 0.3692 ± 0.07735 N = 58; Tumor 4.863 ± 0.1323 N = 511. p < 0.001). **b** Patients with higher PITX2 expression had a relatively lower overall survival. (p = 0.0345). **c** PITX2 was upregulated in 76.67% of lung adenocarcinoma tissues collected from our own hospital (normalized to adjacent normal tissues). **d**–**f** Overexpression of PITX2 correlated with advanced T stage, N stage and TNM stage. **g**, **h** PITX2 mRNA and protein are highly expressed in LUAD cell lines (normalized to HBE, human bronchial epithelial cell) (*p < 0.05, **p < 0.01, ***p < 0.001)

**Table 1:** Correlation between PITX2 expression and clinical pathological characteristics

Characteristics	High level of PITX2 expression (n = 128)	Low level of PITX2 expression (n = 128)	χ^2^	p-value
Age (years)			0.46	0.498701
≤ 60	42	37		
> 60	86	91		
Sex			0.14	0.706625
Male	68	71		
Female	60	57		
Primary tumor			8.74	0.00311*
T1–T2	100	117		
T3–T4	28	11		
Lymph node			0.07	0.788778
N0	88	86		
N1–N2	40	42		
Metastasis			6.61	0.0367*
M0	79	98		
M1	5	3		
MX	44	27		
TNM stage			6.52	0.010652*
I–II	91	108		
III–IV	37	20		

* Significant correlation

### Knockdown of PITX2 inhibited progression of LUAD in vitro

To examine the biological function of PITX2 in LUAD, two siRNAs against PITX2 were transfected into NCIH1299 cell lines. Confirmed by qRT-PCR and western blotting (Fig. 2a), both siRNAs effectively silenced the expression of PITX2 (interfering efficiency, si1 75.3%; si2 75.29%). Furtherly we found that knockdown of PITX2 inhibited proliferation of NCIH1299 cells, validated by CCK-8 assay (Fig. 2b), RTCA assay (Fig. 2c) and colony formation assay (Fig. 2d). Transwell (Fig. 2e) and matrigel (Fig. 2f) assay revealed that knockdown of PITX2 suppressed the migration and invasion ability of LUAD cells. In addition, flow cytometry assay suggested that knockdown of PITX2 induced G1/S cell cycle arrest (Fig. 2g) and TUNEL staining proved that silencing PITX2 led to higher apoptosis ratio of NCIH1299 cells (Fig. 2h).

The article "PITX2 enhances progression of lung adenocarcinoma by transcriptionally regulating WNT3A and activating Wnt/β-catenin signaling pathway" was published in 2019. Journal: Cancer Cell Int.

**Fig. 2:** Knockdown of PITX2 suppressed malignant phenotype of lung adenocarcinoma in vitro. **a** Two siRNAs effectively knocked down the expression of PITX2 in NCIH1299 cell lines (interfering efficiency, si1 75.3%; si2 75.29%). **b**, **c** CCK-8 and RTCA assays showed that knockdown of PITX2 inhibited proliferation of NCIH1299 cell lines. **d** In colony formation assay, NCIH1299 cell lines transfected with si-PITX2 presented less colony count compared with control group (si1, p < 0.001; si2, p < 0.001). **e**, **f** Confirmed by transwell and matrigel assays, knockdown of PITX2 suppressed the migration and invasion ability of NCIH1299 cell lines (si1, p < 0.001; si2, p < 0.001). **g** Knockdown of PITX2 induced G1/S cell cycle arrest in NCIH1299 cell lines (si1, p < 0.001; si2, p < 0.001). **h** TUNEL assay revealed that NCIH1299 cell lines exerted higher apoptosis ratio after knockdown of PITX2 (si1, p < 0.001; si2, p < 0.001) (*p < 0.05, **p < 0.01, ***p < 0.001)

### PITX2 displayed its biological function via activating Wnt/β-catenin signaling pathway

To analyze the signaling pathways associated with PITX2, 317 genes highly co-expressed with PITX2 were used for Gene_Ontology Pathway (Fig. 3a) and Reactome Pathway analysis (Fig. 3b). Results showed that PITX2 might participate in “signal transduction”, “apoptotic process”, “regulation of proliferation” and “gene transcription”. In String database, PITX2 was predicted to interact with LEF1, CTNNB1 and AXIN, all of which are the key factors of Wnt/β-catenin signaling pathway (Fig. 3c). As previous studies have reported that Wnt/β-catenin pathway is regulated by PITX2 in many diseases [18, 37, 38], we performed experiments to test the influence of PITX2 on Wnt/β-catenin downstream genes. It turns out that knockdown of PITX2 significantly downregulated the expression of CCND1, CD44, MYC and JUN on both mRNA and protein levels (Fig. 3d, e). The TOP/FOP flash luciferase assay, a method to examine the activity of Wnt/β-catenin pathway, revealed that reporter expression was suppressed by knockdown of PITX2 (Fig. 3f). And Wnt agonist 1, an activator of Wnt/β-catenin pathway, rescued the effect of PITX2 on proliferation (Fig. 3g) and apoptosis (Fig. 3h) in LUAD cells. These results suggested that the oncogenic role of PITX2 was dependent on Wnt/β-catenin pathway.

The article "PITX2 enhances progression of lung adenocarcinoma by transcriptionally regulating WNT3A and activating Wnt/β-catenin signaling pathway" was published in 2019. Journal: Cancer Cell Int.

**Fig. 3:** PITX2 promoted aggressiveness of lung adenocarcinoma via regulating Wnt/β-catenin signaling pathway. **a**, **b** Gene_Ontology and Reactome Pathway analysis showed that PITX2 might participate in “signal transduction”, “apoptotic process”, “regulation of proliferation” and “gene transcription”. **c** In String Database, PITX2 is predicted to interact with LEF1, CTNNB1 and AXIN, all of which are the key factors of Wnt/β-catenin signaling pathway. **d**, **e** QRT-PCR and western blotting indicated that knockdown of PITX2 decreased the expression of Wnt/β-catenin downstream genes (CCND1, CD44, MYC, JUN) in LUAD cells. **f** Silencing of PITX2 reduced the transcriptional activity of β-catenin while Wnt agonist1, an activator of Wnt/β-catenin pathway, restored the effect. **g** Wnt agonist1 rescued the influence of PITX2 on proliferation in LUAD cells. **h** In TUNEL assay, Wnt agonist1 reversed the increased apoptosis caused by knockdown of PITX2 in LUAD cells (*p < 0.05, **p < 0.01, ***p < 0.001)

### PITX2 regulated the transcription of WNT3A in LUAD cells

It has been confirmed that the encoded protein of PITX2 acts as a transcription factor to regulate gene expression. As shown by Animal TF DataBase, the TF binding site of PITX2 was presented (Fig. 4a). WNT3A, one of the most important ligands in canonical Wnt/β-catenin signaling pathway, has been well established in the progression of LUAD [39–41]. Predicted by hTFtarget website, PITX2 potentially targets the promoter region (1092–1101 bp) of WNT3A (Fig. 4b). Then we constructed luciferase reporter plasmids carrying WNT3A promoter (wild type and mutant type), and luciferase reporter assay revealed that PITX2 increased wild type but not mutant WNT3A promoter luciferase activity (Fig. 4c). Moreover, the results of ChIP assay suggested that PITX2 directly targeted the promoter region of WNT3A (Fig. 4d, e). In NCIH1299 cell lines, knockdown of PITX2 suppressed the expression of WNT3A (Fig. 4f). And in TCGA dataset, PITX2 had a positive correlation with WNT3A (R = 0.22, p < 0.001) (Fig. 4g). These findings indicated that PITX2 controlled the activity of Wnt/β-catenin signaling pathway via transcriptional regulating WNT3A.

**Fig. 4:** PITX2 regulated WNT3A transcription by directly binding to its promoter region. **a** The TF binding site of PITX2 was shown by Animal TF DataBase. **b** Predicted by hTFtarget website, PITX2 directly binds to the promoter region (1092–1101 bp) of WNT3A. **c** Ectopic expression of PITX2 increased wild type but not mutant WNT3A promoter luciferase activity (p < 0.001). **d**, **e** In ChIP assay, PITX2 antibody recruited WNT3A promoter DNA fragment. The IgG antibody and control primer were used as negative controls. **f** The expression of WNT3A were decreased by knockdown of PITX2 (p < 0.001). **g** In TCGA dataset, PITX2 had a positive correlation with WNT3A (R = 0.22, p < 0.001) (Fgiure4G) (*p < 0.05, **p < 0.01, ***p < 0.001)

The article "PITX2 enhances progression of lung adenocarcinoma by transcriptionally regulating WNT3A and activating Wnt/β-catenin signaling pathway" was published in 2019. Journal: Cancer Cell Int.

### Knockdown of PITX2 inhibited tumor growth of LUAD cells in vivo

To investigate the oncogenic role of PITX2 in vivo, xenograft tumor models (six nude mice per group) were used and tumors were harvested at 6 weeks after transplantation (Fig. 5a). The volume and weight of tumors were measured and results showed that tumor growth was significantly suppressed by knockdown of PITX2 (Fig. 5b, c). And immunohistochemistry (IHC) staining with corresponding antibodies revealed that knockdown of PITX2 downregulated the expression of WNT3A, CyclinD1 and C-Myc (Fig. 5d).

**Fig. 5:** Knockdown of PITX2 inhibited proliferation of LUAD in vivo. **a** The tumor xenografts were excised and representative images were shown. **b**, **c** Knockdown of PITX2 suppressed tumor growth and decreased tumor weight in nude mice (n = 6 per group). **d** Immunohistochemical staining showed that knockdown of PITX2 reduced the expression of WNT3A, CyclinD1 and C-Myc (*p < 0.05, **p < 0.01, ***p < 0.001)

### MiR-140-5p was a direct target of PITX2 and suppressed progression of LUAD

To determine the regulatory miRNAs of PITX2, three miRNA prediction datasets were analyzed and the results showed that miR-140-5p potentially bound to PITX2 (Fig. 6a). According to the binding site, luciferase reporter plasmids carrying PITX2 3′UTR (wild type and mutant type) were constructed (Fig. 6b) and luciferase reporter assay showed that ectopic expression of miR-140-5p decreased the luciferase activity of wild type PITX2 3′UTR but not mutant type (Fig. 6c). Furtherly confirmed by qRT-PCR and western blotting, the expression of both PITX2 and WNT3A were down-regulated by ectopic expression of miR-140-5p (Fig. 6d, e). And by transfecting miR-140-5p mimics into NCIH1299 cells, we found that miR-140-5p inhibited tumor proliferation (Fig. 6f), reduced the transcriptional activity of Wnt/β-catenin (Fig. 6g) and induced apoptosis (Fig. 6h) in LUAD cells. Meanwhile, these biological functions of miR-140-5p could be restored by overexpression of PITX2 (Fig. 6f–h). As miR-140-5p played vital roles in LUAD progression, we examined the expression of miR-140-5p in 60 pairs of LUAD tissues. Results revealed that miR-140-5p was significantly down-regulated in LUAD tissues (Fig. 6i) and had a negative correlation with PITX2 (p < 0.0001, R = − 0.5866) (Fig. 6j).

The article "PITX2 enhances progression of lung adenocarcinoma by transcriptionally regulating WNT3A and activating Wnt/β-catenin signaling pathway" was published in 2019. Journal: Cancer Cell Int.

**Fig. 6:** The function of PITX2 in LUAD was inhibited by miR-140-5p. **a** Venn diagram of microRNAs predicted to bind PITX2. **b** MiR-140-5p potentially targets position 135-141 of PITX2 3′UTR and the mutant type of PITX2 3′UTR was constructed. **c** MiR-140-5p decreased the luciferase activity of wild type PITX2 3′UTR but not mutant type (p < 0.001). **d**, **e** Ectopic expression of miR-140-5p reduced the expression of PITX2 and WNT3A in both mRNA and protein level (p < 0.001). **f** MiR-140-5p inhibited proliferation of LUAD cells and PITX2 restored the effect. **g** MiR-140-5p reduced the transcriptional activity of β-catenin (p < 0.001). **h** Confirmed by TUNEL assay, miR-140-5p induced apoptosis of LUAD cells, which can be rescued by PITX2. **i** The expression of miR-140-5p was downregulated in LUAD tissues (relative to paired normal tissues, p < 0.001). **j** The expression of miR-140-5p and PITX2 had a negative correlation (p < 0.0001, R = − 0.5866)

## Discussion

In this study, we found that PITX2 was significantly upregulated in LUAD tissues and correlated with dismal overall survival and advanced clinical stages of patients. Knockdown of PITX2 inhibited tumor growth of LUAD both in vitro and in vivo. And PITX2 exerted its oncogenic role via activating Wnt/β-catenin pathway, especially by regulating the transcription of WNT3A. Furthermore, we found that miR-140-5p was a target of PITX2 and suppressed the progression of LUAD (Fig. 7).

**Fig. 7:** PITX2 plays an oncogenic role in LUAD by transcriptionally regulating WNT3A and thus activating Wnt/β-catenin pathway. And the function of PITX2 can be inhibited by miR-140-5p

The progression of cancer is closely linked to activation of oncogenes and inactivation of tumor suppressor genes [42–44]. LUAD is the most predominant histological subtype of lung cancer and multiple genomic alterations function in cancer growth [45, 46]. The best known is that approximately 15–20% of LUAD harbor epidermal growth factor receptor (EGFR) mutations [47]. However, the functional impact of most genomic alterations of LUAD remains largely unknown. To better understand novel functional genomic alterations in LUAD is hopefully to provide new treatment targets for LUAD patients. As a member of homeobox gene, PITX2 plays a role in the terminal differentiation of somatotroph and lactotroph cell phenotypes [48], is involved in the development of the eye [49], tooth and abdominal organs [50], and acts as a transcriptional regulator involved in basal and hormone-regulated activity of prolactin [51]. Recently, more and more studies show the critical role of PITX2 in many kinds of cancers. In breast cancer cells, upregulation of PITX2 promotes letrozole resistance via transcriptional activation of IFITM1 signaling [52]. The PITX2 DNA methylation was confirmed as a biomarker for the risk and prognosis of colorectal carcinoma [53], head and neck squamous cell carcinoma [54], urothelial bladder cancer [55] and prostate cancer [56]. Increasing researches are showing the significance of development-related genes in cancer progression. KDM5B, a critical regulator during early embryonic development, plays a critical role in controlling stem cell function and tumorigenesis [57]. GREM1, a member of antagonist family that has been shown to relay the sonic hedgehog (SHH) signal from the polarizing region to the apical ectodermal ridge during limb bud outgrowth in mouse, is involved progression of various cancers [58–60]. Similarly, we identified the oncogenic role of PITX2 in LUAD.

The article "PITX2 enhances progression of lung adenocarcinoma by transcriptionally regulating WNT3A and activating Wnt/β-catenin signaling pathway" was published in 2019. Journal: Cancer Cell Int.

In aspect of mechanism, we found that PITX2 promoted LUAD progression as least partially by activating Wnt/β-catenin pathway. Wnt/β-catenin pathway causes an accumulation of β-catenin in the cytoplasm and its eventual translocation into the nucleus to act as a transcriptional coactivator of transcription factors that belong to the TCF/LEF family [61]. Wnt/β-catenin pathway is involved in virtually every aspect of embryonic development and also controls homeostatic self-renewal in a number of adult tissues [62]. Epigenetic dysregulation of Wnt/β-catenin pathway plays a significant role in the pathogenesis of several human cancers [63–65]. The targeting of Wnt protein to the plasma membrane and the binding to its receptor are the initiation process of activating Wnt/β-catenin pathway [66]. As an important member of WNT gene family, WNT3A enhances β-catenin-dependent transcription through GSK3β inhibition or direct β-catenin phosphorylation at Ser^552^ [67]. WNT3A has been reported to promote the migration and invasion process of LUAD and impact prognosis of LUAD patients [41]. And our results suggested that PITX2 directly bound to the promoter region of WNT3A and enhanced its transcription. The oncogenic role of PITX2 is relied on its transcription of WNT3A and thus activating Wnt/β-catenin pathway.

MicroRNAs regulate post-transcriptional gene expression via binding to the 3′UTR of mRNA, and either inhibit protein translation or destabilize target mRNA [21]. Technologies aimed at replacing tumor suppressor miRNA that are lost during cancer progression have emerged as promising cancer therapies [68]. As we have clarified the role of PITX2 in LUAD, to determine the regulatory miRNA of PITX2 is hopefully to provide alternative approach for managing LUAD. Our results revealed that miR-140-5p directly targeted the 3′UTR of PITX2 and suppressed the progression of LUAD. MiR-140-5p has been reported to inhibit progression of many kinds of cancers and regulate the Wnt/β-catenin pathway [69–71]. The miR-140-5p-PITX2-WNT3A axis participates in the regulation of LUAD progression and Wnt/β-catenin pathway, which provides a new sight into the pathogenesis of LUAD.

The article "PITX2 enhances progression of lung adenocarcinoma by transcriptionally regulating WNT3A and activating Wnt/β-catenin signaling pathway" was published in 2019. Journal: Cancer Cell Int.

## Conclusion

To sum up, our study identified PITX2 as a novel oncogene in LUAD. PITX2 promoted progression of LUAD partially by activating Wnt/β-catenin pathway, especially by transcriptional regulating the crucial member of Wnt ligands family, WNT3A. Further research revealed that miR-140-5p directly targeted the 3′UTR of PITX2 and suppressed the progression of LUAD. The miR-140-5p-PITX2-WNT3A axis provides a new sight into the tumorigenesis of LUAD and may represent a potential biomarker and a promising therapeutic target for LUAD patients.

## Additional files

**Additional file 1: Table S1.** 317 genes used for pathway analysis.

**Additional file 2: Table S2.** Sequences of qRT-PCR primers.

**Additional file 3: Table S3.** Sequences of shRNAs and miRNA mimics.

**Additional file 4: Table S4.** Clinical data of 60 LUAD patients.

## Abbreviations

LUAD: lung adenocarcinoma
TCGA: The Cancer Genome Atlas
IHC: immunohistochemistry
ChIP: chromatin immunoprecipitation
UTR: Untranslated Region
